# Factors associated with decision-making power on family planning utilization among HIV-positive women attending public health facilities in Eastern Ethiopia

This article has been retracted.

**DOI:** 10.1186/s40834-022-00175-y

**Published:** 2022-06-02

**Authors:** Hiwot Dejene, Derara Girma, Leta Adugna, Bilisumamulifna Tefera

**Affiliations:** 1 Department of Public Health, College of Health Sciences, Salale University, Fitche, Ethiopia; 2 Department of Public Health, College of Health Sciences, Mettu University, Mettu, Ethiopia

**Keywords:** Women, Decision-making power, Family planning, HIV-positive, ART, Ethiopia

## Abstract

**Background:**

Family planning for HIV-positive women has numerous advantages. However, the need of family planning utilization is challenged by women’s nonautonomous decision-making power. Therefore, this study aimed to examine the level and associated factors of decision-making power to utilize family planning among HIV-positive married women.

**Methods:**

A facility-based cross-sectional study was conducted from March to June 2020 among 363 HIV-positive married women on ART, using systematic random sampling technique. Logistic regression analysis was used to identify variables that affect women’s decision-making power on family planning utilization. Statistical significance was declared at *p*-value < 0.05 with 95% confidence interval and strength of association was reported by adjusted odds ratio.

**Results:**

Overall 55.2% (95% CI: 49.9–60.5) of the women had decision-making power on family planning utilization. Women’s having good knowledge (AOR: 2.87, 95% CI: 1.52–5.40), favorable attitude (AOR: 1.96, 95% CI: 1.13–3.38), women’s getting family planning counseling in ART clinics (AOR: 2.04, 95% CI: 1.16–3.59), women who get integration service of FP and ART (AOR: 1.83, 95% CI:1.07–3.12) were factors independently associated with women decision-making power on family planning utilization.

**Conclusion:**

Decision-making power to utilize family planning among married HIV-positive women was low. Factors like poor knowledge about family planning, dissatisfaction with family planning service, not getting counseling about family planning in ART clinics, and not receiving family planning service in ART clinics were independently associated with women's decision-making power on family planning. Infrastructure linked with the health facility, knowledge, and attitudinal factors should all be combined in future family planning programs.

**Supplementary Information:**

The online version contains supplementary material available at 10.1186/s40834-022-00175-y.

## Introduction

In 2019, worldwide, 38 million people were living with HIV/AIDS [1]. Women of reproductive age are disproportionately affected by HIV/AIDS epidemic. Many HIV-positive women are simultaneously at risk for unintended pregnancy and sexually transmitted diseases (STDs). The utilization of contraception to prevent unintended pregnancy is among the World Health Organization (WHO) recommendations for the prevention of mother to child transmission (PMTCT) of HIV/AIDS [2]. The WHO four-pronged strategy for PMTCT includes reducing the unmet need for family planning (FP) among HIV-positive women and integrating reproductive health /FP and HIV services/ [3]. Consistently, HIV-positive women are expected to benefit from FP services likewise women in the general population, by delaying first births, lengthening birth intervals, and reducing the total number of children born to a woman [4].

The decision-making power of women on family planning is women’s ability to freely decide individually or discuss with their partners family planning needs and choices [5]. Independent decision-making or partners’ communication on family planning utilization has a substantial contribution to the improvement of maternal health [6]. Similarly, ensuring family planning access and allowing women to decide independently to use family planning is important in preventing unintended pregnancy [7].

Women will benefit more from FP if they exercise their human rights to health autonomy and family size decision-making [8]. However, women are often unable to access sexual and reproductive health services due to harmful and discriminatory social norms and practices, lack of agency, and limited financial resources [9]. The majority of women in poor nations do not have access to basic rights [10]. As husbands play a crucial role in FP uptake and avoiding unwanted pregnancies [11], women are subject to collective decision-making by their spouses on reproductive matters [12]. Also, studies indicated that there is a breach in autonomous decision-making power among HIV-positive women to utilize FP [8].

Among HIV-positive women, partner preference is a significant barrier to utilising contraception [13]. In contrast, being able to decide independently/jointly have significance like enhancing other reproductive health decision making [14], increasing utilization of barrier method (condom) [15] and other family planning methods [16]. Besides, the evidence demonstrated that there is a significant association between the contraceptive decision-making process and the integration of services for HIV/AIDS [17].

Various studies conducted among HIV-positive women indicated autonomous decision-making power to utilize FP ranges from 25–80% [18–20]. This suggests that HIV-infected couples faced a serious quandary in making an informed decision to use family planning [21]. This will also result in the underachievement of the planned women's decision-making power at all levels of political, economic, and public life [22]. Nonetheless, no attempts were made in Ethiopia to estimate HIV-positive women's decision-making power regarding FP utilization which will create enormous challenges for planning, implementation, and evaluation of FP activities. Therefore, this study aimed to identify the level of women's decision-making power on FP utilization and associated factors among HIV-positive married women.

## Methods

### Study design, setting, and participants

A facility-based cross-sectional study design was carried out from March 24 to June 12, 2020. The study was carried out at all public health facilities that provide HIV/AIDS care and treatment services, owning anti-retroviral therapy clinics in Dire Dawa city, Eastern Ethiopia. The city is located at 515 km in the east direction of Addis Ababa, the capital city of Ethiopia. Currently, nine health institutions in the city provide ART services (seven health centers, one referral hospital, and one general hospital), and the service is linked with family planning services in all of them. The total HIV-positive married reproductive age (15–49) women attending ART clinics at public health facilities in Dire Dawa city was 2,345. HIV-positive married reproductive age (15–49) women attending ART clinics at public health facilities in Dire Dawa city during the study period and who had at least one previous visit at ART clinics were eligible for the study.

### Sample size determination and sampling techniques

The sample size was calculated using Epi info for estimation of a single population proportion with the assumptions of 95% confidence level, a margin of error (d) of 0.05, and 0.5 prevalence (P) was used due to there was no previously done study on this specific population. Thus, after adding 10% of the non-response rate, the final sample size obtained was 363. Then, the sample size was distributed using proportional allocation to size (PAS) to each ART clinic in the city. A systematic random sampling technique was applied to recruit the study participants. The first participant to be interviewed was selected using the lottery method within the interval. Finally, every six-patient coming to the antiretroviral therapy clinics for a follow-up service had been included until the total sample size was achieved.

### Data collection procedures

Data were collected using a pretested structured questionnaire via face-to-face interview to capture information on socio-demographic characteristics, socioeconomic status of the respondents, reproductive history, knowledge of family planning, attitude towards FP, client satisfaction with the service, and health service-related factors. Medical records were reviewed to get HIV and clinical-related factors. Data were collected by trained nine Bachelor's degree holder nurses that work in the ART clinics and were supervised by two public health officers.

### Measurements

Decision-making power on modern contraceptive use tools has been developed for three sets of women: current users, ever users, and non-users. The developed tool has similar contents which were asked contextually for these sets of women. Each item in the tool has three options (women only, husband only, and joint decision). If the women responded women only and joint decision score of 1 was given, and if the husband only score of 0 was given. Six questions were asked to create a mean score. After computing the total, a score above the mean was considered as having decision-making power [23]. Thus, the tool was highly reliable in the study (Cronbach-alpha = 0.814).

The nine items tool was used to construct a composite score of women’s knowledge about family planning. The first six items have multiple responses and for each response, the score with options “No = 0” and “Yes = 1” was created. The rest of the three questions are based on “Yes = 1” and “No = 0” options. Based on the summation score, a score above 70% was considered as having good knowledge about family planning [24]. Furthermore, the tool has an acceptable reliability test in the current study (Cronbach-alpha = 0.784).

Attitude towards FP was measured by eight Likert scale items. Each item of the question has 5-points ranging from 1 (very unsatisfied) to 5 (very satisfied). A total score was calculated for each domain and transferred into ‘percent score’ by dividing the score with the possible maximum score and multiplying by 100. Those who scored less than 85% were categorized as unfavorable whereas more or equal to 85% as favorable [25]. The tool has an acceptable reliability test in the current study (Cronbach-alpha = 0.854).

Client satisfaction with FP service was measured using fourteen Likert scale items. Each item of the question had 5-points ranging from 1 (very unsatisfied) to 5 (very satisfied) and finally, the mean score was computed to indicate whether or not women were satisfied with the service. To apply the measurement first the woman must be either ever user or a current user [26]. The tool has an acceptable reliability test in the current study (Cronbach-alpha = 0.842).

The wealth index was measured by a simplified and updated Ethiopian wealth index equity tool. The tool contains 15 simplified household assets questions available from www.equitytool.org. The tool has an 84.2% agreement and 0.755 kappa statistics with the full Ethiopian Demographic Health Survey (EDHS,2016) wealth index measurement tool. Accordingly, the wealth index of the household was classified into three groups: poorest, middle and richest [27].

To measure the degree of women's involvement in domestic decision-making, under three subheadings: decisions regarding children (5 items), economic decisions (8 items), and decisions related to social, cultural, and family relations (5 items), were used with options (0 = husband, 1 = wife, 2 = joint). Then, for each subheading, a mean score was computed to classify the presence/absence of involvement in decision making.

Ten Likert scale items were used to measure attitude on gender equity with options (0 = disagree, 1 = Neutral, 2 = Agree). A score above 80% was considered as having a gender-equitable attitude otherwise not an equitable attitude [23].

### Data quality control

The questionnaires were translated to the local language (Amharic language) by a language expert and back-translated to English to guarantee consistency. The one-day training was given to the data collectors on the objective of the study, method of data collection, and ethical issues. The supervisors were also trained on how to monitor the data collection procedures. A pretest was done on 10% of the sample size in Hiwot Fana referral hospital to check the clarity and consistency of the questionnaires before the actual data collection. A reliability test was done and Cronbach-α > 0.7 was taken for actual data collection. During data collection; each completed questionnaire was checked for completeness, clarity, and consistency at the site of data collection by the supervisors to take corrective measures.

### Data processing and analysis

Data were entered into Epi Data version 3.1 and exported into SPSS version 25 for analysis. Data exploration was carried out to assess the completeness and descriptive statistics were used to describe the study participants’ data based on its nature. Binary logistic regression analysis was done for each independent variable with the outcome variable to select candidate variables at a *p*-value < 0.25. Then, entered into multivariable analysis using backward stepwise logistic regression to identify factors associated with the outcome variable and to control for confounders. The adjusted odds ratio with a 95% confidence interval and respective *p*-value < 0.05 was computed to measure the strength of the association and to declare significant variables respectively. Multicollinearity was checked by using VIF and there was no multicollinearity detected at a value of 10. Model fitness was checked by Hosmer & Lemeshow goodness of test (*p*-value = 0.910).

## Results

### Socio-demographic characteristics

A total of 357 married HIV-positive women were participated in this study, with a response rate of 98.3%. The mean (SD) age of the women was 32 (6) years. Regarding the education status, more than three-fourths of the respondents (85.7%) and their husbands (85.1%) have attained formal education. Moreover, more than a third (34.5%) of the respondents were appear in the richest household wealth index class (Table 1).

**Table 1:** Socio-demographic characteristics of married reproductive age HIV-positive women attending ART clinics in Dire Dawa administrative city, Eastern Ethiopia (*n* = 357)

Variables	Categories	Frequency	Percentage
**Age of the respondent**	15–24	47	11.5
	25–34	223	54.5
	35–49	139	34
**Duration of marriage**	< 5 years	42	11.7
	≥ 5 years	315	88.2
**Residence**	Urban	241	67.5
	Rural	116	32.5
**Religion status of the respondent**	Muslim	142	39.7
	Orthodox	134	37.5
	Protestant	75	21.0
	Catholic	6	1.6
**Educational status of the respondent**	No formal education	51	14.3
	Primary level education	105	29.4
	Secondary and above	201	56.3
**Educational status of the husband**	No formal education	53	14.8
	Primary level education	146	40.9
	Secondary and above	158	44.3
**Occupational status of the respondent**	Housewife	130	36.4
	Merchant	74	20.7
	Daily laborer	45	12.6
	Government employee	67	18.8
	Private employee	35	9.8
	Students	6	1.6
**Occupational status of her husband**	Merchant	73	20.4
	Daily laborer	46	12.9
	Government employee	93	26.1
	Private employee	127	35.6
	Others*	18	5.0
**Household wealth index**	Lowest wealth index	115	32.2
	Middle wealth index	119	33.3
	Highest wealth index	123	34.5

*students, farmers

### Client related factors

All study participants had a previous history of using family planning services. Nearly three-fourths of the clients (71.1%) were satisfied with the family planning services. Regarding knowledge and attitude towards FP, near half (45.1%) of the respondents had better knowledge and more than a third (39.2%) of the women had a favorable attitude. Concerning client’s domestic decision-making more than one-third (35.6%) of the women had low involvement in children related decisions, more than half of the respondents (52.6%) had better involvement in the economic-related decision, and only less than one-third (31.6%) of the participants had low involvement in socio-cultural and family relation decision. Regarding gender attitude, only 60.5% of the participants had an equitable attitude (Table 2).

**Table 2:** Client-related factors of married reproductive age HIV-positive women attending ART clinics in Dire Dawa administrative city, Eastern Ethiopia (*n* = 357)

Variable	Categories	Frequency	Percentage
**Knowledge about FP**	Poor	196	54.9
	Good	161	45.1
**Attitude towards FP**	Unfavorable attitude	217	60.8
	Favorable attitude	140	39.2
**Client satisfaction with FP service**	Satisfied	254	71.1
	Dissatisfied	103	28.9
**Domestic decision making**	**Children related**		
	Low involvement	127	35.6
	Better involvement	230	64.4
	**Economic**		
	Low involvement	169	47.3
	Better involvement	188	52.7
	**Socio-cultural & family relations**		
	Low involvement	113	31.7
	Better involvement	244	68.3
**Gender Attitude**	Inequitable attitude	141	39.5
	Equitable attitude	216	60.5

### HIV and health service-related factors

The mean (SD) duration after ART starts was 6.58 (3.61) years. The mean (SD) CD4 count of the respondent was 342 (149.24) cell/mm3 and one-fourth (24.7%) of them were found in severe immune suppression. Only 9.5% of the respondents undisclosed their HIV status to their partner (Table 3). Few more than half (53.8%) of the respondents not received integration FP service in the ART clinics. In contrast, nearly two-thirds (65.5%) of the respondents were received FP counseling service in the ART clinics (Fig. 1).

**Table 3:** HIV-related factors of married reproductive age HIV-positive women attending ART clinics in Dire Dawa administrative city, Eastern Ethiopia (*n* = 357)

Variables	Categories	Numbers	Percentage
**Duration of ART started**	≤ 3 years	85	20.8
	> 3 years	323	79.2
**Partner tested**	Yes	305	85.4
	No	26	7.3
	I don’t know	26	7.3
**Disclosure status**	Yes	322	90.2
	No	35	9.8
**Partner HIV status**	Positive	243	68.1
	Negative	62	17.4

**Fig. 1:** Health service-related factors of married reproductive age HIV-positive women attending ART clinics in Dire Dawa administrative city, Eastern Ethiopia (*n* = 357)

### HIV-positive women decision-making power on family planning

The level of decision-making power on family planning among married HIV-positive women was 55.2% (95%CI: 49.9%-60.5%) (Fig. 2).

**Fig. 2:** Women decision making power on family planning among of married reproductive age HIV-positive women attending ART clinics in Dire Dawa administrative city, Eastern Ethiopia (*n* = 357)

### Factors associated with woman decision making power on family planning

Bivariable analysis showed that sociodemographic variables (age of the respondent, educational status of the husband), client-related factors (knowledge about family planning, attitude towards family planning, and client satisfaction with family planning service), HIV related factors (duration on ART, partner HIV status and disclosure status) and health service-related factors (counseling service in ART service and integration of FP service with ART) were a candidate for multivariable analysis. In multivariable logistic regression analysis: The odds of FP using decision-making power were more than twice greater among women who had good knowledge about FP than those who had poor knowledge about FP (AOR = 2.06, 95%CI:1.25–3.39). The practice of decision-making power on FP use was two times more common among women who had a favorable attitude towards family planning than their counterparts (AOR = 1.96, 95%CI:1.13–3.38). The odds of decision-making power on FP use among women who get counseling service in ART clinics were two times higher than the odds of decision-making power on FP use among women who do not get counseling service at the same place (AOR = 2.04, 95%CI:1.16–3.59). The current study also revealed that HIV-positive women who receive integrated FP and ART services were almost two times more likely to practice decision-making power than those who do not receive integrated FP and ART services (AOR = 1.83, 95%CI:1.07–3.12) (Table 4).

**Table 4:** Factors associated with women decision-making power on family planning among HIV positive married women attending ART clinics in Dire Dawa administrative city Eastern Ethiopia (*n* = 357)

Variable	Categories	Women decision making power on FP		COR (95% CI)	AOR (95% CI)
		Yes (%)	No (%)		
Age of the respondent	15–24	19 (46.3)	22 (53.7)	1	1
	25–34	115 (59.6)	78 (40.4)	1.70 [0.867–3.36]	1.29 [0.51–3.26]
	35–49	63 (51.2)	60 (48.8)	1.21 [0.59–2.46]	1.49 [0.86–2.58]
Educational status of the husband	No formal education	26 (49.1)	27 (50.9)	1	1
	Primary education	71 (48.6)	75 (51.4)	0.98 [0.52–1.84]	0.97 [0.46–2.09]
	2^nd^ & above education	100 (63.3)	58 (36.7)	1.79 [0.95–3.35]	1.15 [0.54–2.47]
**Knowledge about FP**	**Poor**	**86 (43.9)**	**110 (56.1)**	**1**	**1**
	**Good**	**111 (68.9)**	**50 (31.1)**	**2.84 [1.83–4.39]**	2.06 [1.25–3.39] **
**Attitude towards FP**	**Unfavorable attitude**	**108 (49.8)**	**109 (50.2)**	**1**	**1**
	**Favorable attitude**	**89 (63.6)**	**51 (36.4)**	**1.76 [1.14–2.72]**	1.96 [1.13–3.38] *
Client satisfaction	Satisfied	157 (61.8)	63 (61.2)	2.54 [1.59–4.08]	1.31 [0.76–2.24]
	Dissatisfied	40 (38.8)	97 (38.2)	1	1
Duration on ART	≤ 3 years	37 (48.7)	39 (51.3)	1	1
	> 3 years	159 (56.8)	121 (43.2)	1.38 [0.83–2.30]	1.41 [0.76–2.61]
Partner HIV status	Positive	144 (59.3)	99 (40.7)	1.45 [0.83–2.54]	1.64 [0.89–2.99]
	Negative	31 (50.0)	31 (50.0)	1	1
Disclosure status	Yes	186 (57.8)	136 (42.2)	2.98 [1.41–6.29]	1.30 [0.29–5.65]
	No	11 (31.4)	24 (68.6)	1	
**counseling in ART**	**Yes**	**151 (64.5)**	**83 (35.5)**	**3.045 [1.93–4.79]**	2.04 [1.16–3.59] *
	**No**	**46 (37.4)**	**77 (62.6)**	**1**	**1**
**Integration of FP and ART service**	**Yes**	**113 (68.5)**	**52 (31.5)**	**2.79 [1.81–4.32]**	1.83 [1.07–3.12] *
	**No**	**84 (43.8)**	**108 (56.2)**	**1**	**1**

^**^ significant at *p*-value < 0.001

^*^ significant at *p*-value < 0.05

1 = references

## Discussion

Women's empowerment has been reported to be central to the use of family planning [28]. In developing countries, the majority of partners offer women inferior roles in all areas of decision-making [23, 28, 29]. As a result, women are either involved in joint decision-making with their husbands and/or dependent solely on the decision of the male partner on matters concerning their use of contraceptives and reproductive life [30]. In this study, the magnitude of HIV-positive women's decision-making power in family planning was 55.2%. This result is consistent with a study done among uninfected women in Dinsho woreda [31]. The comparability might be due to both studies being conducted among married women.

However, the current finding is lower than a study done among uninfected women in Gedeo zone and Dawro [5, 23]. This discrepancy might be due to the difference in socioeconomic, demographic status, and population background of married women. Furthermore, this is because infected women may be more vulnerable to rights abuses than uninfected individuals. Besides, male-dominated reproductive decision-making is a major challenge for HIV-infected women [32].

In contrast to the above, this finding is higher than the results from Ethiopian DHS 2016 [33]. In the current study, having regular medical attention and being exposed to frequent counseling from a health care practitioner may boost decision-making capability. Furthermore, the disparity might be attributable to differences in research settings, since the current study was conducted at facility levels as opposed to the EDHS, which was community-based. Similarly, our finding is higher than the study conducted in Adwa, Ethiopia [34]. The reason for this might be related to time change, which could improve women's empowerment and men's understanding of women's reproductive health rights.

This study also examined factors associated with women's decision-making power on family planning use. Accordingly, having good knowledge of family planning was associated with decision-making power in family planning use. This result is supported by the study done among uninfected women in southern Ethiopia [23]. This might be due to women who have better knowledge of contraceptives will develop autonomy to use/discuss with their partners about family planning. Moreover, women who have a favorable attitude towards family planning were more likely to decide on family planning use than women who have unfavorable attitudes. This is supported by studies done among uninfected women in southern Ethiopia [5, 23, 31]. The findings show the practical role attitudes play in guiding decision-making.

This study also revealed that women who get counseling services from health personnel to use family planning methods in ART clinics were more likely to have decision-making power on family planning than women who do not get counseling services from a health professional in ART clinics. This might be due to counseling being important to help women and their partners to gain increased control over their reproductive health. It also increases FP uptake, and continuation is essential for ensuring informed and voluntary decision making [35]. HIV-positive women who receive integrated family planning services with ART had more decision-making power in family planning than women who do not receive integrated services. This is because support from the health system during integrated service will facilitate decision-making power [36].

### Limitation of the study

The cross-sectional nature of the study design does not allow causality ascertainment.

## Conclusion

This study shows married HIV-positive women had low decision-making power on FP use according to the national demographic health survey [37]. Factors that increase women's risk of having low decision-making power on FP use were poor knowledge about FP, dissatisfaction with FP service, women do not receive counseling on FP in ART clinics, and women do not take FP service in ART clinics. Therefore, promoting FP knowledge and improving attitudes toward FP are keys to rise women’s decision-making power to utilize family planning. Furthermore, FP programs could also support HIV-positive women receiving FP counseling during ART clinic visits and make integrated FP services more accessible in ART clinics. Besides, applying a mixed-method approach in future studies in this regard will be beneficial to understanding influencing factors of decision-making power on FP use.

## Supplementary Information

**Additional file 1.**

**Additional file 2.**

## Data Availability

The data used in this study will be issued from corresponding author based on reasonable request.

## Abbreviations

AIDS: Acquired Immuno-Deficiency Syndrome
ART: Antiretroviral Therapy
EDHS: Ethiopian Demographic Health Survey
FP: Family Planning
HIV: Human Immuno-deficiency Virus
PMTCT: Prevention of Mother to Child Transmission
STD: Sexually Transmitted Diseases
WHO: World Health Organization
